The article "Occupational Dysfunction as a Mediator between Recovery Process and Difficulties in Daily Life in Severe and Persistent Mental Illness: A Bayesian Structural Equation Modeling Approach" was published in 2022. Journal: Occup Ther Int.

# Occupational Dysfunction as a Mediator between Recovery Process and Difficulties in Daily Life in Severe and Persistent Mental Illness: A Bayesian Structural Equation Modeling Approach

**DOI:** 10.1155/2022/2661585

**Published:** 2022-06-17

**Authors:** Aki Watanabe, Takayuki Kawaguchi, Mai Sakimoto, Yuya Oikawa, Keiichiro Furuya, Taichi Matsuoka

**Affiliations:** ^1^Department of Rehabilitation, Kitasato University School of Allied Health Sciences, Sagamihara City, Kanagawa, Japan; ^2^Department of Community Mental Health and Law, National Institute of Mental Health, National Center of Neurology and Psychiatry, Kodaira City, Tokyo, Japan; ^3^Link Yokohama Home-Visit Nursing Station, Yokohama City, Kanagawa, Japan; ^4^Minori Home-Visit Nursing Station Yurigaoka, Kawasaki City, Kanagawa, Japan; ^5^Department of Recovery Support, Fukui Memorial Hospital, Miura City, Kanagawa, Japan

## Abstract

**Background:**

This study is aimed at verifying a hypothetical model of the structural relationship between the recovery process and difficulties in daily life mediated by occupational dysfunction in severe and persistent mental illness (SPMI).

**Methods:**

Community-dwelling participants with SPMI were enrolled in this multicenter cross-sectional study. The Recovery Assessment Scale (RAS), the World Health Organization Disability Assessment Schedule second edition (WHODAS 2.0), and the Classification and Assessment of Occupational Dysfunction (CAOD) were used for assessment. Confirmatory factor analysis, multiple regression analysis, and Bayesian structural equation modelling (BSEM) were determined to analyze the hypothesized model. If the mediation model was significant, the path coefficient from difficulty in daily life to recovery and the multiplication of the path coefficients mediated by occupational dysfunction were considered as each the direct effect and the indirect effect. The goodness of fit in the model was determined by the posterior predictive *P* value (PPP). Each path coefficient was validated with median and 95% confidence interval (CI).

**Results:**

The participants comprised 98 individuals with SPMI. The factor structures of RAS, WHODAS 2.0, and CAOD were confirmed by confirmatory factor analysis to be similar to those of their original studies. Multiple regression analysis showed that the independent variables of RAS were WHODAS 2.0 and CAOD, and that of CAOD was WHODAS 2.0. The goodness of fit of the model in the BSEM was satisfactory with a PPP = 0.27. The standardized path coefficients were, respectively, significant at −0.372 (95% CI: −0.586, −0.141) from “difficulty in daily life” to “recovery” as the direct effect and at −0.322 (95% CI: −0.477, −0.171) mediated by “occupational dysfunction” as the indirect effect.

**Conclusions:**

An approach for reducing not only difficulty in daily life but also occupational dysfunction may be an additional strategy of person-centered, recovery-oriented practice in SPMI.

## 1. Introduction

The concept of recovery is becoming increasingly central to mental health policy and support services internationally. However, confusion and challenges remain in exploring the meaning of recovery and reflecting it in support practices for individuals with severe and persistent mental illness (SPMI). The definition of recovery has been described as “a way of living a satisfying, hopeful, and contributing life even with limitations caused by illness” [1]. Recovery encompasses “clinical recovery” (i.e., symptom reduction and functional recovery) and “personal recovery” (e.g., regaining hope, taking control and responsibility for one's life, participating in social roles and meaningful activities, and redefining one‘s identity), and this classification contributes to the understanding of the concept [2, 3]. In particular, personal recovery is primarily about restoring the right of people with SPMI to live safe, dignified, personally meaningful, and satisfying lives in the community while having a mental illness [4]. This recovery movement is to be welcomed because it brings optimism about the possibility of healing and of engaging in a process of change in a person's relationship to distress for individuals with SPMI [5]. The components of personal recovery described in the systematic review and narrative synthesis conducted by Leamy et al. [6] were organized and structured into a framework comprised of the following: Connectedness, Hope & optimism, Identity, Meaning, and Empowerment. This framework with the acronym CHIME has been widely endorsed and has contributed greatly to recovery-oriented evaluation, practice, and research as an evidence base for respecting the understanding that recovery is a unique and individual experience rather than something the mental health system does to a person [6, 7]. However, highlighting only the optimistic aspects of recovery has led to criticism and suspicion of fostering individualism in that individuals are responsible for difficult experiences resulting from poor policies and support services [5, 8]. Therefore, recovery-oriented practices for individuals with SPMI require a more expansive understanding of the individual's subjective experience in the recovery process.

A useful finding for a broader understanding of people's recovery experiences to implement a personalized recovery-oriented practice seems to have involved the relationship to “difficulties.” Through a systematic review and best-fit framework synthesis with the CHIME framework, Stuart et al. [9] proposed the inclusion of D, indicating “difficulties,” as a component of recovery in the CHIME framework to extend the recovery concept. The literature suggested that “difficulties” mainly refers to ambivalence, disempowerment, negative life changes, and conflicts and that these are a major part of the recovery process [9]. In addition, a clearer understanding of to what extent difficulties are contextually dependent was contended as being valuable in ascertaining how services can assist people with SPMI [9]. Recently, some surveys were conducted to understand the actual situation of difficulties in people with SPMI using large-scale data. A recent study using the World Health Organization Disability Assessment Schedule second edition (WHODAS 2.0) [10], which assesses difficulties experienced in activities of daily living, suggested that gender, age, education, economic status, medical hospitalization, and unemployment were factors of difficulty in the daily life of people with schizophrenia [11]. One research report found that the employment status of people with schizophrenia can be determined by the cut-off score of WHODAS 2.0 [12]. These reports indicate that difficulties in daily life are dependent on the context of the individual with SPMI and also influence the context of the individual. However, to reflect these findings into a person-centered approach, a structural understanding is needed to answer the following research question: How do the subjective experiences of people affected by a disability that arise in life processes play a role between recovery process and difficulties in daily life? To address this issue, we decided to conduct an empirical study using generalized measurement tools to examine the causal structure of the recovery process and difficulties in daily life, including the subjective experiences of individuals. Occupational dysfunction with a theoretical background in the model of human occupation was adopted to investigate in detail the individual's subjective experiences related to difficulties in daily life [13]. Occupation in this paper refers not only to its work-related meaning (including business, employment, and labor), but also to the natural biological system of health symbolized by “doing,” “being,” and “becoming” (including education, play, activities of daily living, rest, and social participation) [14]. Therefore, occupational dysfunction is defined as a condition in which a person is unable to properly perform activities of daily living and is a major health-related problem that has evolved primarily in the field of preventive occupational therapy [13, 15]. A patient-reported outcome measure (PROM) was developed that can be categorized into four-factor categories (i.e., occupational marginalization, occupational imbalance, occupational alienation, and occupational deprivation) that contribute to an understanding of the subjective state when people experience occupational dysfunction [15]. Occupational marginalization is defined as when a person does not have the opportunity to engage in desired daily activities [15, 16]. Occupational imbalance is defined as a loss of balance in engaging in daily activities [15, 16]. Occupational alienation is defined as a situation in which the inner needs of the individual related to daily activities are not satisfied [15, 16]. Occupational deprivation is defined as a lack of opportunity for daily activities beyond the individual's control [15, 16]. Previous studies in occupational dysfunction have shown it to be a factor associated with psychological problems in stress response, burnout syndrome, and depression in health care workers [17, 18]. In addition, the relationship of occupational dysfunction to health-related quality of life in undergraduate students or metabolic syndrome and its component factors in community-dwelling Japanese adults has also been examined [15, 19]. However, the relationship between occupational dysfunction and the recovery process in people with SPMI has yet to be examined. In several Japanese practical studies of support services for people with SPMI, individualized service planning and collaborative practice based on occupational dysfunction have been reported [15, 20]. Therefore, forming and assessing a hypothesis that would be possible to construct a structural model of the recovery process and difficulties in daily life including occupational dysfunction as a factor are necessitated.

A clearer understanding of an individual's recovery process may require a complex approach to the construction of personal narratives and meanings [21]. By assessing the causal structure of the recovery process and difficulties in daily life including occupational dysfunction, the significance of this study is to show that service providers should be concerned with and address the meaning of the difficulties in an individuals' recovery process. Although empirical research on the relationship of health-related concepts to the recovery process among individuals with SPMI is needed, it is not yet fully implemented. We formed a hypothetical model that includes both the direct effect of “difficulties in daily life” to “recovery process” without mediating variables and the indirect effect of “difficulties in daily life” to “occupational dysfunction” to “recovery process” via mediating variables (see Figure 1). Analysis based on Bayesian structural equation modelling (BSEM) was adopted to examine the effectiveness of the mediating variables. Indirect effects are significant when occupational dysfunction plays an important role between the recovery process and difficulties in daily life. Therefore, the purpose of this study was to examine the factor structure of the recovery process and difficulties in daily life, including occupational dysfunction as a health-related indicator for persons with SPMI.

## 2. Materials and Methods

### 2.1. Participants

Participants in this multicenter cross-sectional study were community-dwelling individuals with SPMI responding to recruitment between April to August 2017 and November 2017 to March 2018 in 21 community facilities. The facilities included 7 psychiatric daycare facilities, 5 outpatient occupational therapy facilities, supportive residential care facilities (4 group homes and 1 life training facility), 3 home-visit nursing stations, and 1 employment support facility.

Although there are several definitions of SPMI [22–24], the National Institute of Mental Health's definition was adopted for its comprehensiveness [25]. The study was restricted to individuals who had been diagnosed as having schizophrenia, major depression, or bipolar disorder for at least two years because this study included individuals with mixed ICD-10 or DSM-5 diagnostic criteria for which details were not available. The eligibility criteria were (i) individuals who are 20 years old or older and continue to receive outpatient care, (ii) individuals with confirmed severe episodes because it was assumed that some of the individuals would have a mild dysfunction in the Global Assessment of Functioning (GAF) by using the current services, and (iii) individuals who could understand the questionnaire and give their consent to the explanation of this study. The details of severe episodes included a previous hospitalization, unemployment status, and status of the need for daily living support due to frequent use of services in a week. Individuals with a diagnosis of organic psychotic disorders were excluded. Although this was a low-risk and noninvasive study, individuals with symptom instability and/or confusion were excluded to reduce the burden of participation in this study.

### 2.2. Procedure

The data of gender, age, period of education, diagnosis category, duration from diagnosis, and the GAF score were collected from the medical records as individual factors. In each facility where the GAF score was not recorded, experienced research collaborators assessed the GAF score using a modified-GAF scale with other professionals at the same time as data collection [26, 27]. The services and their frequency of use, family members, and current employment were collected from medical records or the subject's description. The assessment used the Japanese version of the Recovery Assessment Scale (RAS) [28], the WHODAS 2.0 [29], and the Classification and Assessment of Occupational Dysfunction (CAOD) [15] as the means of subjective assessment.

### 2.3. Assessment Scales

#### 2.3.1. RAS

The RAS is the pioneering and most widely used self-reported scale for assessment of the recovery process in people with mental illness [30, 31]. The reliability and validity of the 24-item RAS used in this study have been previously validated in Japan [28]. The 24-item RAS consists of items related to the five recovery factors of “goal/success orientation and hope,” “reliance on others,” “personal confidence,” “no domination by symptoms,” and “willingness to ask for help.” Participants were asked to answer 24 questions on a 5-point Likert response scale ranging from 1 (strongly disagree) to 5 (strongly agree). The total score range is 24–120. The total score for each item was calculated, with a higher total score indicating high orientation in the recovery.

#### 2.3.2. WHODAS 2.0

The WHODAS 2.0 is a comprehensive rating scale developed by WHO as a tool for assessing one's activity limitations and participation constraints and for measuring difficulties in daily life activities as a disability based on the International Classification of Functioning, Disability and Health (ICF) [10, 29]. In this study, the 36-item self-completion version was used. The WHODAS 2.0 assesses an individual's level of functioning in six major life domains: (i) cognition (understanding and communication); (ii) mobility (ability to move and get around); (iii) self-care (ability to attend to personal hygiene, dressing, and eating and to live alone); (iv) getting along (ability to interact with other people); (v) life activities (ability to carry out responsibilities at home, work, and school); and (vi) participation in society (ability to engage in community, civil, and recreational activities). Participants were asked to answer 36 questions on a 5-point Likert response scale ranging from “no problem” to “I can't do anything at all.” Standardized scores were used for each domain and the total score. The score range is 0–100 for both the total score and the score in each major life domain. Higher scores indicate more difficulties in daily life based on health problems.

#### 2.3.3. CAOD

The CAOD is an assessment of occupational dysfunction as a condition in which a person is unable to perform living activities properly [15]. It includes four domains (occupational imbalance, occupational deprivation, occupational alienation, and occupational marginalization) in which a person feels limited in the activities of living [13, 15]. The participants were asked to answer 16 questions on a 7-point scale from “1 (disagree)” to “7 (agree).” The score range was 16–112, and higher total scores indicate more severe occupational dysfunction.

### 2.4. Analysis

Confirmatory factor analysis for each scale was adopted to measure the structural validity of the three assessments, and reliability coefficients were analyzed. A model with the corresponding subitems influenced by each factor and covariance assumed among all factors was created, and the goodness-of-fit index was obtained. The subitems of each scale were considered based on the standardized estimates, GFI (goodness-of-fit index), AGFI (adjusted GFI), and RMSEA (root mean square error of approximation), and the internal consistency of each scale was confirmed by calculating Cronbach's alpha coefficient. The standardized estimate for the deletion of items was less than 0.5. An acceptable goodness of fit of >0.85 [32] or >0.90 [33] for GFI, >0.85 [32] or >0.95 [33] for AGFI, and RMSEA is considered <0.08 to be an acceptable upper limit [34]. However, we adopted >0.85 for GFI and AGFI because this study used clinical data and included participants in a variety of services. Moreover, Spearman's rank correlation coefficient was performed to examine latent variables that should be considered for addition in the hypothetical model. Multiple regression analysis by the forced entry method was determined to estimate covariates involved in the hypothetical model and to clarify their causal relationships with the variables that showed a significant relationship in the correlation as the independent variables and “RAS,” “WHODAS 2.0,” and “CAOD” as the dependent variables. Based on these results, we planned to verify the hypothesized model of the recovery process and difficulties in daily life mediated by occupational dysfunction. Even though the required sample size was 161 or more for power = 0.8 and *α* = 0.05 in structural equation modelling (SEM) [35], we decided to adopt the BSEM approach that accommodates smaller sample sizes [36]. To analyze whether the statistical power for the acceptable goodness of fit index RMSEA = 0.08 [37], the sample size of the collected data, *α* = 0.05, and the degree of freedom (df) in the SEM were sufficient, a post hoc power analysis was performed using the “semPower” package in the statistical software R [38]. If the causal model was significant, the path coefficient from difficulties in daily life to the recovery process was considered a direct effect, and the multiplication of the path coefficient from difficulties in daily life to occupational dysfunction and from occupational dysfunction to the recovery process was considered an indirect effect. The Markov chain Monte Carlo method was conducted for BSEM estimation. The goodness of fit in the model was assessed by the posterior prediction method and the posterior predictive *P* value (PPP). A PPP > 0.10 was considered to indicate a good model fit [39]. The path coefficients and 95% confidence intervals between the latent variables in the model were also analyzed. The path coefficient was considered to be significant when the 95% confidence intervals did not contain zero. The set number of sampling times was 100,000, and the algorithm was considered to have converged when the convergence statistic was less than set 1.002.

Statistical analyses were conducted using SPSS Statistics 27 software (IBM, USA), SPSS Amos ver. 25.0 (IBM, USA), and R (version 4.1.2), and a *P* value of <0.05 was considered statistically significant.

### 2.5. Ethics Statement

This study was approved by the Kitasato University Medical Ethics Organization (KMEO B16-200) and each facility. The purpose and content of the study were explained, and written informed consent was obtained from each participant. We also explained that participation in this study was voluntary and that participants would incur no disadvantage even if participants did not agree or withdrew their consent.

## 3. Results

### 3.1. Characteristics of the Participants

The characteristics of the participants are shown in Table 1. The participants comprised 98 community-dwelling individuals (55 males and 43 females) with a mean age of 50.4 ± 11.2 years. Clinical categories included schizophrenia (70 cases, 71.4%), major depression (17 cases, 17.3%), and bipolar disorder (11 cases, 11.2%), and duration from being diagnosed was 20.9 ± 10.6 years. Eighty-eight patients (89.8%) had experienced hospitalization one or more times. The duration of the current service use other than outpatient care was 57.0 ± 59.7 months. The current service use facility was psychiatric daycare in 52 cases (53.1%), which is more than half, and included participants who were forced to use supportive residential care (18 cases, 18.4%). Sixty-four participants (65.4%) used the current service more than three times a week, and most of the week was spent using the services. In addition, none of the participants who required outpatient treatment and service use worked in competitive employment. The assessment for each evaluation scale is shown in Table 2. In the RAS, the total score was biased toward the higher side of the score range. In the WHODAS 2.0 and CAOD, the total score and each domain were biased toward the lower side of the score range.

### 3.2. Relationship between each Assessment Scale

A confirmatory factor analysis was conducted on the subitems of each assessment scale. The standardized estimates of each subitem ranged from 0.51 to 0.93. The GFI, AGFI, and RMSEA values, which indicate the goodness of fit of the model, were, respectively, 0.840, 0.774, and 0.045 for the RAS, 0.790, 0.734, and 0.038 for the WHODAS 2.0, and 0.916, 0.867, and 0.000 for the CAOD, and the RAS, WHODAS 2.0, and CAOD were confirmed to have a five-, six-, and four-factor structures, respectively. Cronbach's alpha for each scale was 0.911 for the RAS, 0.930 for the WHODAS 2.0, and 0.918 for the CAOD. Spearman's rank correlation analysis, conducted to identify latent variables to consider adding to the hypothetical model, showed a moderately significant correlation among the scales (see Table 3). In addition, to clarify the causal relationship between each variable, a multiple regression analysis using the forced entry method was conducted with “RAS” and “CAOD” as the dependent variables and the independent variables as those showing significant correlations with each other. The independent variables for “RAS” were the total score of the WHODAS 2.0 and the CAOD (coefficient of determination: *R*^2^ = 0.404, *P* < 0.001) and that for “CAOD” was the total score of the WHODAS 2.0 (*R*^2^ = 0.284, *P* < 0.001) (see Table 4). The multiple regression analysis for the dependent variable “WHODAS 2.0” was rejected as no variables with significant correlation.

### 3.3. Causal Structure of Recovery Process, Difficulties in Daily Life, and Occupational Dysfunction

The result of post hoc power analysis in SEM showed that a sample size of *N* = 98 was associated with a power = 92.1% to reject a wrong model (with df = 74) with an amount of misspecification corresponding to RMSEA = 0.08 on *α* = 0.05. From the above results, the causal factors affecting the recovery process were hypothesized to be “difficulties in daily life” and “occupational dysfunction” affecting “recovery process,” and a hypothetical model of causality in the recovery process was developed (see Figure 1), following which BSEM was used. The latent variables were “recovery process,” “difficulties in daily life,” and “occupational dysfunction,” and the observed variables were the scores on the subitems of each factor. The convergence statistic for Bayesian estimation was 1.001, which was stable. The PPP was 0.27, which was better than 0.10, indicating a satisfactory value. The standardized path coefficients [95% confidence interval] between latent variables in the BSEM were 0.598 [0.419, 0.731] from “difficulties in daily life” to “occupational dysfunction,” −0.539 [−0.734, −0.310] from “occupational dysfunction” to “recovery process,” and −0.372 [−0.586, −0.141] from “difficulties in daily life” to “recovery process” (as the direct effect), all of which were significant. The indirect effect from “difficulties in daily life” to “recovery process” mediated by “occupational dysfunction” was −0.322 (0.598 × −0.539), and the 95% confidence interval was [−0.477, −0.171] (see Figure 2).

## 4. Discussion

As one of the few quantitative studies based on PROM in community-dwelling individuals with SPMI using mental health services, the present study was conducted to examine the relationship between the recovery process and difficulties in daily life. Participants in this study included those with mild global functional impairment (as indicated by the GAF) due to long-term treatment and service use. However, all participants had experienced severe episodes of illness, such as hospitalization or unemployment, that required some service use in addition to outpatient care. Many participants were still using services multiple times per week and continued to be unemployed or in partial or sheltered employment and had difficulty achieving financial independence. This study was unique in its examination of the hypothesis of whether occupational dysfunction as an individual's subjective health-related indicator could be a factor between the two latent variables of the recovery process and difficulties in daily life in individuals with SPMI. According to the result of the BSEM, its structure was a mediation model showing the direct effect of difficulties in daily life on the recovery process and the indirect effect through occupational dysfunction as a mediating factor. The goodness of fit in the model was satisfactory, with moderate and similar direct and indirect effects on the recovery process from difficulties in daily life, respectively. Specifically, the direct effect indicated that the recovery process for individuals with SPMI was hindered by increasing difficulties in daily life. This result supported previous research that suggested that the components of recovery should include difficulties [7, 9]. The indirect effect indicated that the greater the occupational dysfunction as a subjective experience resulting from difficulties in daily life, the more inhibited was the recovery process. Conversely, the model indicated that reductions of difficulties in daily life or occupational dysfunction could directly facilitate or indirectly support the recovery process impeded by difficulties in daily life. This visualization of the model based on the recovery process and difficulties in daily life has not been used much when examining recovery-oriented approaches, even though it could represent a person-centered approach. The previous studies seemed to have been biased toward those that focused primarily on the relationship between the recovery process and objective levels of disability or symptoms [40, 41]. However, the difference between personal and clinical recovery stems from the fact that clinicians and clients were concerned with different aspects of mental illness [7]. Thus, our study was designed to bridge the gap between clinicians and clients by visualizing the structural relationship between the recovery process and difficulties in daily life as indicating the need to address subjective experiences such as occupational dysfunction in individuals with SPMI. Moreover, the factor structure of each PROM in individuals with SPMI in this study was confirmed to be similar to the original studies in other populations, which allowed us to capture the desired phenomenon [10, 15, 28, 29]. The results indicated a part of the validity of using each PROM adopted for individuals with SPMI and provided basic information for comparison with other populations.

In this study, other data except for difficulties in daily life and occupational dysfunction were not adopted as additional factors in the hypothetical model during the analysis phase. First, in this regard, the correlation between the recovery process and global functioning was not significant. This result is different from a previous review that indicated a low correlation between the recovery process and global functioning [42]. However, the results of the present study support this review, which considers whether the global functioning indicated by the GAF scored by clinicians may not reflect important aspects of functioning from the people's perspective [42]. This might have been affected by relatively mild functional impairment in community life, as the participants' inherent functional status was masked by the long-term use of mental health services. Other than the above, there was no correlation between difficulties in daily life as a subjective level of disability and global functioning as in a previous study [43]. In addition, even though there was a low correlation between occupational dysfunction and global functioning, the causal relationship was not significant. Furthermore, although demographic data such as age and level of education were crucial factors of difficulties in daily life in a previous study [11], they were not included as relevant factors in the present study. Despite the limited information with different sample sizes, it was interesting to note that the items surveyed were not identified as any additional factors influencing the structural relationship between the recovery process and difficulties in daily life. Previous studies suggested that objective assessments were not always consistent with subjective assessments [44, 45]. Personal recovery is subjective by definition, and thus, it is reasonable to attempt to capture it by subjective measurement rather than objective one. The model validated in this study potentially emphasized the importance of capturing the subjective state, including the meaning of difficulties, rather than the presence or absence of difficulties only, when clinicians approach clients' difficulties in daily life for the personal recovery of their clients. However, even though the demographic data and objective measures we examined in this study remain potentially detectable in larger sample sizes, they might not be significantly relevant for inferring the meaning of difficulties for individuals with SPMI.

The present model suggested the practical implications of a recovery-oriented approach based on the difficulties in daily life for individuals with SPMI. Specifically, there were two approaches to the recovery process: a direct approach to reducing the difficulties in daily life for individuals with SPMI and an indirect approach to improving the meaning expressed in the occupational dysfunction resulting from their difficulties. Inherently, personal recovery is not intended to be a clinical outcome but rather a process that involves both difficulties and opportunities to overcome them and is routinely considered a deeply personal experience [7, 46]. There was a need for “more personalized” PROMs that can reflect the subjective experiences associated with recovery for people with SPMI [47]. Our findings were based on including the result of a PROM of occupational dysfunction defined as the inability to function in an occupation that was central to human experience (i.e., what one should do, wants to do, and is expected to do) and attempting to capture seriously the structural relationship between the recovery process and difficulties in daily life [14–16]. People with SPMI facing stigma, trauma, and poverty might struggle to agree on the positive aspects of personal recovery presented in CHIME [7]. In this regard, “occupational alienation,” “occupational deprivation,” “occupational imbalance,” and “occupational alienation” included in occupational dysfunction were negative experiences in a person's daily life and indicated subjective “meanings” resulting from difficulties [15, 17]. The shared understanding of the meaning between the client and the clinician is essential to the collaborative process of establishing goals and care plans to address the client's difficulties [48]. Subjective meanings resulting from difficulties can be captured and shared through PROM-based interviews, even though they may be unnoticed by the individuals and are easily latent. Capturing and sharing the meaning of the difficulties influenced by the individual's life background and environmental factors with them would lead to a personalized recovery-oriented approach and assistance for their recovery process. In other words, when alienation, deprivation, imbalance, and marginalization occur in the face of challenges that are difficult for the client to directly alleviate, the client and the clinician can begin to collaborate by thinking together to improve those meanings of difficulties. An approach based on the model including occupational dysfunction would be expected to bridge the gap between clients (subjective) and clinicians (objective) in how they perceive the difficulties of clients with SPMI and to promote meaning-making as a step toward beginning to collaborate toward the recovery process [49]. Therefore, the findings of this study supported the expanded CHIME-D (including “D: difficulties”) proposed by Stuart et al. [9] and would be suitable as a model embodying an approach to meaning arising from difficulties for the recovery process of persons with SPMI.

The strength of this study is that it is the first study, to our knowledge, to validate the structural relationship between the recovery process and difficulties in daily life by including occupational dysfunction as a mediating factor in individuals with SPMI. The first of several limitations is that this study was biased to indicators of life impact areas adopted in internationally influential systematic reviews because it focused on the structural relationship between the recovery process and the difficulties in daily life [50]. Even though the GAF assesses a global functional state that encompasses mental and social functioning [42], the severity of symptoms, and the amount of medication were not investigated. Second, although as much demographic data as possible were collected, it was difficult to collect any information on income and regional characteristics that have been identified as factors causing difficulties in daily life in large-scale surveys in Asia [11]. Adding such information to the closed mediation model obtained in this study could be extended to multilevel structural equation modeling and provide further information that contributes to a recovery-oriented approach by a more realistic and extensive model. Third, there were concerns about whether the results could be generalized to areas under different insurance systems because the participants in this study used services based on the Japanese insurance and mental health systems. Fourth, the participants in this study were individuals who were accustomed to using either community mental health care or services and were volunteers who responded to recruitment. The study did not include individuals who were slightly affected by the degree of difficulty in building a relationship with the clinicians due to just starting to use the services and potential service users who still lived in the community. The characteristics of the SPMI population selected for this study affected the relatively high level of the recovery process in the results of the RAS and biased the milder difficulties in daily life and occupational dysfunction in the WHODAS 2.0 and CAOD. This may be the reason why the desired GFI and AGFI for each scale were not yielded in the confirmatory factor analysis [32, 33]. For example, the skewed scores in each domain typified by “Self-care” of WHODAS 2.0 reflect the impact of service use, and the current population did not seem to have much difficulty in daily life with service used depending on the type of activity domains. In contrast, we decided that the RMSEA value of less than 0.06 [51], which is ideal, was an acceptable goodness of fit and continued the analyses. Therefore, there were selection biases that need to be carefully considered about whether the insights gained from this model could be generally applied. In this study, although the present model of the recovery process and the difficulties in daily life were analyzed by including participants from various mental health services, it was necessary to emphasize the limitation that the results were based on the assumption of service use. The fifth limitation to consider is that the results might have been influenced by the recovery-related assessment measures used. Recent studies have debated whether the RAS can adequately assess the recovery process [52, 53]. Although the RAS was recommended among several recovery-related assessment measures, other measures might or might not be suggested to be suitable for assessment based on the CHIME framework [54]. In addition, the RAS had been suggested to be a rating scale that focuses specifically on empowerment among the components of CHIME [55]. Although the present structural relationship was significant because difficulties in activity engagement as a mediator of recovery were considered [56], it was unclear whether similar results would be obtained using recovery-related assessment measures other than the RAS. Finally, although we relied on the minimum sample size required to build the structural equation model in this study, validation with a larger sample size was necessary to increase the statistical power. Adopting the BSEM approach was sufficiently valid to address this point.

## 5. Conclusions

This empirical research study has shown the structural relationship of difficulties in daily life towards the recovery process mediated by occupational dysfunction in individuals with SPMI. The present model was significant as a model of the need to collaborate concretely between clients and clinicians to decrease the negative effects of an overly optimistic view on the recovery process and difficulties in daily life by capturing the meaning of difficulties as they were. This finding did not negate optimism but emphasized the need for a comprehensive understanding of the positive aspects presented in CHIME and the negative aspects of difficulties in daily life in the recovery process of people with SPMI. The occupational dysfunction was shown to be a mediating factor indicating the importance of a person-centered recovery-oriented approach that addresses not only directly alleviates difficulties in daily life but also the subjective aspects resulting from them. In addition, these direct and indirect approaches to difficulties in daily life seemed to have a similar effect on the recovery process. These series of results demonstrated the clinical implications of simultaneously assessing different aspects of personal recovery and recovery-related assessment measures when understanding an individuals' recovery process [40]. Despite the limited information, an assessment of occupational dysfunction as a subjective meaning resulting from difficulties caused by the interaction between the person and life or the environment was recommended. Thus, further research would be required to examine the factors surrounding recovery for properly capturing the recovery process in people with SPMI. The expected future investigation would be based on a longitudinal study to examine whether coping with difficulties in daily life could affect changes in the recovery process.

## Figures and Tables

**Figure 1:** The hypothesis model. A hypothetical model of recovery process in severe and persistent mental illness (SPMI) includes the direct effect of “difficulties in daily life” to “recovery process” without mediating variables, and the indirect effect of “difficulties in daily life” to “occupational dysfunction” to “recovery process” via mediating variables.

**Figure 2:** Structural relationship between the recovery process and difficulties in daily life mediated by occupational dysfunction using Bayesian structural equation modeling. The values in this figure indicate the standardized path coefficients (95% confidence interval).

**Table 1:** Characteristics of the participants.

Characteristic	Value
Participants [*n*]	98
Male/female [*n*]	55/43
Age [years (range)]	50.4 ± 11.2 (22–77)
Period of education^a^ [years (range)]	13.4 ± 2.5 (9–23)
Marital status (married/divorced/not married/bereaved) [*n*]	14/18/62/4
Residence status (living with family/living alone/shared residence) [*n*]	35/39/24
Diagnosis (schizophrenia/major depression/bipolar disorder) [*n*]	70/17/11
Duration from diagnosis^b^ [years (range)]	20.9 ± 10.6 (3–51)
Number of hospitalizations^c^ [*n* (range)]	3.1 ± 3.1 (0–19)
Hospitalization experience (one or more times/none) [*n*]	88/10
Duration of current service use other than outpatient care [months (range)]	57.0 ± 59.7 (0.1–331.8)
Current service use facility (DC/RC/OT/HV/ES) [*n*]	52/18/14/12/2
Frequency of current service use per week (every day/5–6/3–4/1–2/once or less) [*n*]	18/21/25/29/5
Current employment status (PT/SW/UJ/NE/RE) [*n*]	8/17/12/55/6
GAF score [median (interquartile range)]	61.0 (54.0–74.0)

Values are the mean ± standard deviation (range), n or median (interquartile range). ^a^*n* = 94 (due to inclusion of 4 unknown data); ^b^*n* = 95 (due to inclusion of 3 unknown data); ^c^*n* = 97 (due to inclusion of 1 unknown data); DC: psychiatric daycare; RC: supportive residential care; OT: outpatient occupational therapy; HV: home-visit nursing; ES: employment support; PT: employed in a part-time job; SW: sheltered working; UJ: unpaid job (including housework); NE: no employment; RE: retired; GAF: Global Assessment of Functioning.

**Table 2:** Assessment scores.

Assessment	Score
RAS (range of score)	
Personal confidence (5−25)	14.7 ± 3.9 (5–24)
Willingness to ask for help (4−20)	14.3 ± 2.4 (7–20)
Goal and success orientation (9−45)	30.2 ± 6.3 (16–44)
Reliance on others (4−20)	14.2 ± 2.9 (5–20)
No domination by symptoms (2−10)	6.8 ± 2.1 (2–10)
Total score (24−120)	80.1 ± 14.2 (41–112)
WHODAS 2.0 (range of score: 0−100)	
Cognition	25.9 ± 20.3 (0–80)
Mobility	19.5 ± 22.3 (0–81)
Self-care	9.6 ± 15.5 (0–70)
Getting along	34.7 ± 24.6 (0–92)
Life activities	30.8 ± 26.1 (0–100)
Participation in society	32.6 ± 21.9 (0–83)
Total score	27.1 ± 17.7 (0–77)
CAOD (range of score)	
Occupational imbalance (4−28)	10.9 ± 6.0 (4–28)
Occupational deprivation (3−21)	8.9 ± 5.2 (3–21)
Occupational alienation (3−21)	10.4 ± 5.3 (3–21)
Occupational marginalization (6−42)	16.5 ± 8.1 (6–40)
Total score (16−112)	46.7 ± 19.9 (16–110)

Scores are the mean ± SD (range). RAS: Recovery Assessment Scale; WHODAS 2.0: WHO Disability Assessment Schedule 2.0; CAOD: Classification Assessment of Occupational Dysfunction.

**Table 3:** Correlations between variables.

Variables	CAOD	WHODAS 2.0	Age	Period of education^a^	Duration from diagnosis^b^	Number of hospitalizations^c^	Duration of current service use	GAF
RAS	−0.623^∗∗^ (<0.001)	−0.476^∗∗^ (<0.001)	0.004 (0.965)	−0.092 (0.378)	0.101 (0.332)	−0.001 (0.995)	0.173 (0.089)	0.067 (0.510)
CAOD	—	0.497^∗∗^ (<0.001)	−0.134 (0.188)	0.144 (0.167)	−0.068 (0.510)	0.096 (0.347)	0.022 (0.833)	−0.228^∗^ (0.024)
WHODAS 2.0	—	—	−0.044 (0.668)	−0.068 (0.513)	−0.073 (0.483)	0.059 (0.565)	0.002 (0.986)	−0.193 (0.057)

Values are Spearman's correlation coefficient (*P* value). ^a^*n* = 94 (due to inclusion of 4 unknown data); ^b^*n* = 95 (due to inclusion of 3 unknown data); ^c^*n* = 97 (due to inclusion of 1 unknown data); CAOD: Classification Assessment of Occupational Dysfunction; WHODAS 2.0: WHO Disability Assessment Schedule 2.0; GAF: modified Global Assessment of Functioning; RAS: Recovery Assessment Scale. ^∗^*P* < 0.05,  ^∗∗^*P* < 0.01.

**Table 4:** Causal relationships between variables.

Objective variable	Explanatory variable	Partial regression coefficient	Standardized partial regression coefficient (*P*-value)	Adjusted *R*^2^ (*P*-value)
RAS	CAOD	−0.333	−0.467^∗∗^ (<0.001)	0.404^∗∗^ (<0.001)
	WHODAS 2.0	−0.210	−0.261^∗∗^ (0.006)	
CAOD	WHODAS 2.0	0.576	0.511^∗∗^ (<0.001)	0.284^∗∗^ (<0.001)
	GAF	−0.178	−0.119 (0.178)	

Values are the result of a multiple regression analysis by the forced entry method. RAS: Recovery Assessment Scale; CAOD: Classification Assessment of Occupational Dysfunction; WHODAS 2.0: WHO Disability Assessment Schedule 2.0; GAF: modified Global Assessment of Functioning. ^∗∗^*P* < 0.01.

## Data Availability

The data used to support the findings of this study are available from the corresponding author upon request.
